This article has been retracted.

# Computational Intelligence Approaches in Developing Cyberattack Detection System

**DOI:** 10.1155/2022/4705325

**Published:** 2022-03-18

**Authors:** Mohammed Saeed Alzahrani, Fawaz Waselallah Alsaade

**Affiliations:** College of Computer Science and Information Technology, King Faisal University, P.O. Box 4000, Al-Ahsa, Saudi Arabia

## Abstract

The Internet plays a fundamental part in relentless correspondence, so its applicability can decrease the impact of intrusions. Intrusions are defined as movements that unfavorably influence the focus of a computer. Intrusions may sacrifice the reputability, integrity, privacy, and accessibility of the assets attacked. A computer security system will be traded off when an intrusion happens. The novelty of the proposed intelligent cybersecurity system is its ability to protect Internet of Things (IoT) devices and any networks from incoming attacks. In this research, various machine learning and deep learning algorithms, namely, the quantum support vector machine (QSVM), k-nearest neighbor (KNN), linear discriminant and quadratic discriminant long short-term memory (LSTM), and autoencoder algorithms, were applied to detect attacks from signature databases. The correlation method was used to select important network features by finding the features with a high-percentage relationship between the dataset features and classes. As a result, nine features were selected. A one-hot encoding method was applied to convert the categorical features into numerical features. The validation of the system was verified by employing the benchmark KDD Cup database. Statistical analysis methods were applied to evaluate the results of the proposed study. Binary and multiple classifications were conducted to classify the normal and attack packets. Experimental results demonstrated that KNN and LSTM algorithms achieved better classification performance for developing intrusion detection systems; the accuracy of KNN and LSTM algorithms for binary classification was 98.55% and 97.28%, whereas the KNN and LSTM attained a high accuracy for multiple classification (98.28% and 970.7%). Finally, the KNN and LSTM algorithms are fitting-based intrusion detection systems.

## 1. Introduction

The Internet of Things (IoT) could be defined as interlinked systems that focus on standardized mechanisms that communicate large amounts of data [1] between Internet-connected machines. Artificial intelligence (AI), or the quality of being smart, is being introduced to gadgets, devices, houses, businesses, and maybe even communities as a result of the current innovations in IoT. IoT is considered one of the most rapidly evolving disciplines of present technology advancement, contributing significantly to a variety of domains ranging from agriculture to self-driving cars. Because it interacts with each and every form of linked system in everyday life, IoT is known as the use of Internet through everything that can help people in their daily lives.

Fundamental firewalls are static defense systems that act as channels. They are not fit for perceiving an attack. They generally obstruct all traffic with the exception of the packets coordinating a few guidelines; for example, packets are bound to a specific port or originate from the secure Internet Protocol (IP) addresses. These rules are constructed physically by the system overseer as indicated by the network security approach. This implies that the productivity of a firewall relies on how talented the administrator is [2].

The quantity of smart interconnected devices is expected to reach 1 billion in 2025 [2]. IoT is made up of numerous layers, which includes a specific layer called the network layer. The architecture of the network layer depends on the Internet, which is based on different communication layers, and is primarily capable of sending network packets among servers. Furthermore, the network layer is a complicated and vulnerable component of the IoT structure that contributes to a variety of security problems.

Nonetheless, a number of security mechanisms exist to solve security concerns[3]. To enable a set of connected devices to function successfully and address security issues, these mechanisms must be installed in the IoT ecosystem and/or endpoints. However, many security devices require a significant amount of computing power and storage space [4]. To address these limitations, several techniques, including lightweight cryptography and authentication processes, can be used [5]. The vast number of sensors, nodes, servers, or machines associated and interlinked through the IoT architecture is indeed a major source of security concern, as a security incident in either a single node or sensor might cause the entire system to collapse. Cyberattacks, distributed denial-of-service (DDoS) hacks, ransomware, distant monitoring, packet-forwarding attacks, and privacy breaches are by far the most prevalent security vulnerabilities that IoT systems confront. A firewall is generally the first point of security against intrusions in IoT devices, although this is not an efficient option due to the wide range and complication of IoT infrastructures. Intrusion detection systems (IDSs) have risen in importance as a result of its reliability. In 1980, Spafford and James [6] offered a description of an IDS for the very first time. IDSs are designed to detect intrusions in a certain network domain. An intrusion through an IoT context can become a host that attempts to access neighboring nodes without taking permission. An IDS has three major components: a client, a screening test, and a reaction module. The client is entirely accountable for managing data from the tracking actions data stream. The intrusion prevention mechanism detects evidence of intrusion and delivers alarms. Then, the reaction module can be activated using the results that the analysis engine provides. IDSs have improved in reliability and efficiency over time, but hackers have created more diverse attack tactics to circumvent these tracking systems. Furthermore, typical IDSs are incapable of dealing well with IoT's numerous network elements, such as interconnected layers [7].

Researchers have been urged to use decentralized IDSs in addition to different machine learning techniques, including artificial neural networks (ANNs), deep learning, and optimization algorithms, because of recent advances in intelligent machines. Typical ANNs are limited in their ability to cope with the complications of IDS systems. Enhanced technology by addressing such limitations is necessary for IDSs to achieve their potential. The major objective of this paper is to apply blockchains to a multi-agent system and to evaluate its performance using a benchmarking dataset [8, 9].

The main contribution of this study is to apply various machine learning and deep learning algorithms to detect intrusion intelligently. A smart IDS can help to protect the IoT environment from any updated attacks. The system has the ability to detect and prevent cyberattacks in IoT networks. In this study, we investigate various machine learning and deep learning to detect attacks with binary and multiple classes to determine the performance of each model. The network dataset has many network features that obstruct the IDS system from quick detection, enabling the selection of significant features that can help the system save time with a high detection rate. In this study, we use the correlation method to find features that have a significant relationship with classes. Finally, different AI algorithms are investigated to improve the performance and efficiency of IDS systems.

## 2. Related Work

Although the techniques of the Internet of Things are essential for enhancing real-world intelligent systems, such as applications used in smart cities, home automation, and smart factories, and their massive scale and omnipresence have presented unique security concerns [10, 11]. Additionally, because IoT systems are typically used in an uncontrolled environment, an intruder with malevolent aims may gain access to these systems [12, 13]. Snooping can sometimes be employed to get confidential details from such a transmission medium, since IoT components are generally interconnected across wireless networks [14, 15]. Due to their limited power and computing capabilities, IoT-connected devices may not have installed advanced security measures to address the upper edge of such security concerns. Specific attack interfaces emerge on something like a constant basis as a result of the IoT's complexity and interrelated settings [16, 17].

As a result, particularly in contrast to typical computing systems, IoT networks are much more exposed. To mitigate threats faced by IoT-connected devices, appropriate diagnostic and preventive strategies must be developed. Furthermore, a line of defense in distributed systems must be established to defend IoT systems from cyberattacks. IDSs are used to solve this problem [18, 19]. Machine learning-based IDSs that provide security for IoT networks or exploited IoT systems have been reported in many studies. IDSs that are implemented in cloud-based IoT networks [20], sensor networks [21, 22], cyber-physical applications [20], and wireless mobile networks [23, 24] have all been covered by the literature. Classical IDS approaches, on the other hand, are much less efficient or effective for the provision of security networks due to their unique attributes, such as limited power, pervasiveness, diversity, constrained bandwidth utilization, and global connectivity, as noted above. Deep learning and machine learning-based approaches have recently found traction for detecting cyber threats, particularly those affecting IoT networks. This is due to the fact that machine learning- and deep learning-based approaches may detect both benign and malignant abnormalities in an IoT network.

To discover the characteristics of patterns, IoT servers and network flow can be monitored and examined. Any divergence from all learned norms can be leveraged to spot abnormal activity and unusual behavior. Moreover, technologies based on machine learning and deep learning have been used to predict unknown or zero-day cyberattacks. As a result, machine learning- and deep learning-based techniques provide reliable security measures for IoT devices and systems. Several studies have investigated various strategies for developing IDSs for IoT applications, but the majority of the abovementioned surveys did not include the adoption of machine learning or deep learning approaches, such as detection methods in IoT networks and associated compact components. The focus of several studies [25–30] was on investigating IoT security challenges broadly and their categorization in different layers related to applications, networks, cryptography, and access restrictions. An inclusive study that provides a comprehensive evaluation of machine learning and deep learning algorithms that can be adopted in IDS applications in IoT network settings is still needed, as is a key emphasis of this work.

The researchers in [31] focused on the problems with IoT security somewhere within the network layers. A study published in [32] investigated IDS technologies for IoT networks. A preliminary examination of machine learning's applicability in the domain of IoT confidentiality and protection was addressed in [33]. Furthermore, they highlighted bandwidth limitations, processing power limitations, and a lack of suitable space as obstacles in applying any machine learning-based security mechanisms for IoT interconnected systems. Other studies [34, 35] explored the possibility of using machine learning and data mining algorithms to identify malicious attacks and intrusions in IoT networks by incorporating these algorithms in IDSs and recognizing abnormalities or using network data classification. The authors in [20] pointed out differences among IDSs that operate on cellular broadband and wireless communication networks, particularly IoT networks. Due to basic architectural differences, applying machine learning approaches to IoT IDSs involves special attention to the details of cyberattacks, supporting protocols (including both telecommunications and networking), and the application layer. A further study reported in [21] explored how IDSs can be implemented in mobile ad hoc networks. Three major kinds of IDS layouts can be used in mobile ad hoc networks (MANETs). A layered architecture is the first layout that is organized with several hierarchical layers. For deployment in a decentralized and collaborative setting, the second architectural is also flattened. The third layout can be a combination of the first two employed in mobile agents. An additional study [22] explored a number of intrusion detection techniques for mobile ad hoc-based IDS architectures. These IDS techniques, as per the authors, can indeed be divided into several classified methods based on the basic principles employed to identify an intrusion. Rules, metrics, optimizations, signatures, contexts, popularity scores, or pathways can always be utilized as principles in IoT systems. Anomaly discovery, exploitation, signature-based algorithms, and evolutionary algorithms were eventually included in the list of hybrid technologies.

Other classification criteria have been proposed as well [22]. For example, these include real-time/offline, attack type, and effectiveness of detection (scalability, reliability, timeliness, etc.). Other authors provided further classification criteria, such as legitimacy, intrusion patterns, and identification efficacy (scalability, reliability, timeliness, etc.) [22]. In a different study, the author discussed a categorization of IDS for wireless sensor networks (WSN) depending on the IDS agent's configuration model [29]. The configuration model might be decentralized, centralized, or mixed, with the last model being recommended as the ideal fit for WSNs. A similar survey presented in [30] categorized WSNs relying on IDS by utilizing IDS detecting class criteria. Outlier detection, abuse detection, and recognition based on configuration were among the categories discovered. A further facet of the virtualized IoT ecosystem was examined and described in [15] in which the authors of this study evaluated and categorized several cloud-based IDSs that influence the confidentially, authenticity, and reliability of cloud computing that depend on IoT networks. Hypervisor-based IDS, host-based IDS (HIDS), network-based IDS (NIDS), and scalable IDS were all discussed as well. The authors in [29] introduced a research study on IoT-based IDS and specifically focused on IDS design. They looked at current IoT standards, protocols, and solutions, as well as IoT privacy concerns and detecting categories, before proposing an IoT IDS design. In [36], the authors presented a new multiphase anomaly identification technique based on Boruta Firefly aided partitioning density-based spatial clustering of applications with noise (BFA-PDBSCAN). Furthermore, they assumed that their suggested approach provided better experimental results in matching the specified methods of density-based spatial clustering of applications with noise (DBSCAN) and hierarchical density-based spatial clustering of applications with noise (HDBSCAN).

The researchers in [37] presented an integrated data processing approach for outlier identification and classification that incorporates grey wolf optimization (GWO) and convolutional neural network (CNN) algorithms. The researchers stated that their method outperformed existing state-of-the-art IDSs in terms of effectiveness and detection accuracy. A sophisticated autoencoder-based anomaly detector system was utilized to analyze and diagnose IoT botnet intrusions [38]. The approach involved obtaining statistical properties from behavior snapshots of typical IoT edge device data patterns and developing a deep learning-based autoencoder just on extracted features from the used dataset. Furthermore, the reconstruction of errors for traffic measurements was matched to a threshold to determine whether they are normal or abnormal. The authors assessed the suggested identification approach using the BASHLITE and Mirai botnets dataset created with the help of industrial IoT systems.

## 3. Materials and Methods

Figure 1 displays the formwork of the proposed system for detecting intrusion from a real dataset.

### 3.1. Dataset

The KDD Cup dataset was employed to investigate our proposed system. The NSL-KDD is an updated version of the KDD Cup dataset proposed by McHugh [39]. Furthermore, each record consists of 41 features, and these features can be described as either normal or attacks. The KDD Cup and NSL-KDD datasets contain three major intrusions, namely, denial-of-service (DOS), probe, root to local (R2L), and user to root (U2R).  Table 1 demonstrates the feature names for the KDD Cup dataset.

Furthermore, the attack types of the KDD Cup datasets are clustered into four different attack classes: (1) DoS, which includes attacks that cause the slowing or shutting down of a machine by sending more traffic information to the server than the system is able to handle. DoS attacks affect legitimate network traffic or access to services; (2) R2L includes attacks that provide illegal local access to a machine by sending remote deceiving packets to the system; (3) U2R includes attacks that provide root access, and in this case, the hacker finds out the system vulnerability and starts using the system as a normal user; and (4) probe includes attacks that can avoid security control systems by gathering information about the network. The attack categories of the KDD Cup are reported in Table 2.

### 3.2. Preprocessing

The processing method was applied to select significant features from the dataset.

#### 3.2.1. One-Hot Encoding

One-hot encoding was proposed to convert categorical features, namely, protocol type, service, and flag, into numerical features. One-hot encoding is used to assign each string to a new binary value [0, 1].  Table 3 shows the categorical features of both datasets.

#### 3.2.2. Normalization Method

After transforming the categorical features, the data were processed using min-max normalization methods for normalizing the data to avoid overlap in the training process that can occur when handling the largest dataset. In the normalization method used to scale the dataset in the same range, we put the scaling range of data between 0 and 1.

(1) $$\begin{array}{c} z_{n}=\frac{x-\text{y}}{x_{-}y}\left(x_{i}-y_{i}\right)+y_{i}, \end{array}$$

where *y* and *x* are the minimum and maximum data, respectively. The maximum range is represented by *y*_*i*_, whereas the minimum range is indicated by *x*_i_ [0].

#### 3.2.3. Feature Selection Method

Correlation analysis was used to find correlations between the features and classes. It is also used to find significant patterns between features of datasets for intrusion detection.

(2) $$\begin{array}{c} R=\frac{n\sum^{}\left(x\;\times y\right)-\left(\sum x\right)\left(\sum y\right)}{\;\left[n\sum \left(x^{2}\right.\right)-\sum \;\left.\left(x^{2}\right)\right]\;\times \;\left[n\sum \left(y^{2}\right.\right)-\sum \;\left.\left(y^{2}\right)\right]}\times 100\%, \end{array}$$

where *R* is Pearson's correlation coefficient approach, *x* is input training, and *y* is target (classes). We considered the threshold value to be 0.50, the features with a greater-than-0.50 relationship with classes were selected, and everything else was excluded.  Table 4 shows the selected features among 41 features of the KDD Cup datasets. According to the results of the correlation analysis method, the same_srv_rate had a high correlation among 75% all features; therefore, we considered these features as significant.

### 3.3. Classification Algorithms

In this section, the classification algorithm is presented.

#### 3.3.1. Support Vector Machine (SVM)

The support vector machine (SVM) is a prevalent supervised nonlinear technique that can be applied to distribute data sequentially and nonsequentially for classification tasks. SVM is used for text classification, image processing, and anomaly analysis. Furthermore, it has the ability to deliver good accuracy for high-dimensional vector space data and symbolizes data training features in space maps. The data features of the several classes are distinguished based on a maximum margin in the hyperplane. The decision boundary that can be achieved by the SVM technique is represented by the extreme margin space for determining the distance between the training samples of two or more classes. The equation for the SVM classifier is given as follows:

(3) $$\begin{array}{c} K\left(X,X^{\prime }\right)=exp\left(-\frac{\|X-X\prime {\|}^{2}}{2\sigma {\;}^{2}\;}\right), \end{array}$$

where *X*, *X*′ is the feature vector for the training of the evaluated dataset, ‖**X** − **X**′‖^2^ denotes the squared Euclidean difference among two feature inputs, and *σ* is a free parameter.

#### 3.3.2. KNN Algorithm

When the KNN algorithm is adopted for the classification task, it performs the classification of various feature values by computing the distance between each pair. An integer number not more than 20 usually specifies the *k* parameter in this algorithm. While working on the KNN algorithm, the decided neighbors can be represented by various objects that have been accurately identified and categorized. This technique only identifies the class of the sample and can be based on the class of the neighboring one or various samples in the decision making regarding categorization. KNN is utilized to determine the *k* values, which are near a set of values through the training dataset, and the majority of these *k* values fall to a confirmed class; furthermore, the input sample is classified. The equation that was applied for the KNN algorithm is written as follows:

(4) $$\begin{array}{c} \sqrt{\left(x_{1}-x_{2}\right)+\left(y_{1}-y_{2}\right)}. \end{array}$$

The *k* value is utilized to find and calculate the nearest points in the feature vectors. As such, the value must be distinctive.

#### 3.3.3. Long Short-Term Memory (LSTM)

Hochreiter and Schmidhuber [40] proposed the long short-term memory (LSTM) approach for learning long-term information interdependence. An LSTM's flow is similar to that of the recurrent neural network (RNN) method. The difference in how the cells are operated between the LSTM and RNN approaches is that there are four gates in each LSTM unit, specifically the input, candidate, forget, and output gates. The forget gate determines whether data should be saved or destroyed. The cells are refreshed by the input gate, while the output gate always determines the hidden state in the LSTM. The LSTM also has an incorporated memory block and gate mechanism that allows it to resolve vanishing gradient point problems and disintegration gradient complications through the RNN learning process [41, 42]. The structure of the LSTM technique is expressed in Figure 2.

The computing equations that are associated with the LSTM structure in Figure 1 are as follows:

(5) $$\begin{array}{c} \;f_{t}=\sigma \;\left(W_{f\;}.X_{t}+W_{f}.h_{t-1}+b_{f}\right),\\ i_{t}=\sigma \left(W_{i}.X_{t}+W_{i\;}.h_{t-1}+b_{i}\right),\\ S_{t}=\text{tan }h\left(W_{c}.X_{t}+W_{c\;}.h_{t-1}+b_{c}\right),\\ \;C_{t}=i_{t}{\;}^{*}\;S_{t}+f_{t}{\;}^{*}\;S_{t-1},\\ o_{t}=\sigma \left(W_{o}+X_{t}+W_{o}.h_{t-1}+V_{o}.C_{t}+b_{o}\right),\\ h_{t}=o_{t}+\text{tan h}\left(C_{t}\right). \end{array}$$

The mathematical symbolization in the above equations can be interpreted and expressed as follows:

*X*_*t*_ is the vector of the input data that progress to the memory cell at time *t*. *W*_*i*_, *W*_*f*_, *W*_*c*_, *W*_*o*_, and *V*_*O*_ are the weight matrices. *b*_*i*_*b*_*f*_, *b*_*c*_, and *b*_*o*_ represent bias vectors. *h*_*t*_ is the specified value of the memory cell at time *t*. *S*_*t*_ and *C*_*t*_ are the defined values of the candidate state of the memory cell and the state of the memory cell at time *t*, individually.

*σ* and tanh are the activation functions in the LSTM network.

*i*_*t*_, *f*_*t*_, and *o*_*t*_ are acquired values for the input gate, the forget gate, and the output gate at time *t*. These gates have values in the range of 0 to 1 over the nonlinear sigmoid activation function.

#### 3.3.4. Deep Autoencoder Algorithm

Encoders and decoders are two primary components of an autoencoder technique. An encoder component reduces the dimensionality of input data into the lowest dimensional exemplification form, while the decoder reproduces input data depending on the lowest data representation, which is made by the encoder component. Autoencoders, on the other hand, automatically encode all data of the input layer and forward these data into hidden layers before finally decoding the data into the production layer (output layer) in the network [43–47]. Considering the efficiency of autoencoders in discovering different sorts of attacks, the recognition accuracy of an autoencoder-based deep learning model for IDSs might be highly dependent on the nature of the autoencoder model's design and hyperparameter configurations. As a result, finding ideal settings of autoencoders that can lead to better detection accuracy is crucial. Earlier mainstream studies described individually obtaining the right model by running several tests with specific datasets. Human procedure testing takes a long time in intrusion detection tasks, and they must be performed whenever data are updated [48–52]. The deep autoencoder (DAE) model for IDSs achieved through two processes can handle the IoT network security problem. These processes are training and testing [53, 55]. The system utilizes a training dataset to generate a classifier obtained by the selected DAE. In the testing process, an IDS uses the autoencoder model to recognize the class of each sample in the testing dataset to evaluate the overall performance of the system when it can be applied to an online environment.  Figure 3 illustrates the suggested DAE structure for intrusion detection that consists of three different layers: the input, hidden, and output layers.

### 3.4. Performance Measures

The performance measures were used to test the outcomes of the proposed model. Accuracy, false positive, precision, true positive, and time were used. The equations for performance measures are as follows:

(a) Accuracy
  (6) $$\begin{array}{c} \text{accuracy}=\frac{TP+TN}{TP+FP+FN+TN}\times 100\%, \end{array}$$
(b) Precision
  (7) $$\begin{array}{c} \text{precision}=\frac{TP}{TP+FP}\times 100\%. \end{array}$$
(c) F-score
  (8) $$\begin{array}{c} F-\text{score }=\frac{2*\text{precision}*\text{sensitivity}}{\text{precision}+\text{sensitivity}}\times 100\%, \end{array}$$
where TN represents true negative, TP represents true positive, FP represents false positive, and FN represents false negative.

## 4. Experimental Results

This section describes the experimental analysis of the proposed model developed during the research phase. Two experiments were conducted to improve the IDS. The experiment was conducted and evaluated by utilizing the KDD Cup dataset. Python programming language was used to implement all machine learning and deep learning algorithms to design the model. The Jupyter platform was used to run all code. In this study, two experiments were prepared to classify and identify intrusions from the IoT platform.

### 4.1. Results of Binary Classification

In this section, machine learning and deep learning algorithms are proposed to classify intrusion as normal or attacks.

#### 4.1.1. Machine Learning Algorithm with Binary Classification

In this experiment, binary classifications, namely, QSVM, KNN, linear discriminant, and quadratic discriminant algorithms, were applied to detect intrusion. The binary classifications included two classes (normal and attack packets).  Figure 4 shows the instance values of KDD Cup data for normal and attack classes.

The dataset was divided into 70% for training and 30% for testing, and the testing dataset was processed to validate the machine learning algorithms. The evaluation metrics accuracy, precision (%), recall, and F1 score were employed to examine the proposed algorithm to classify intrusion.  Table 5 shows the results of the machine learning algorithms. The KNN algorithm achieved high accuracy (98.55%). The quadratic discriminant algorithm obtained lower accuracy (68.91%). Based on these results, we confirmed that the KNN algorithm is an appropriate algorithm for binary classification.

The statistical metrics to find the prediction errors, namely, MAE, MSE, RMSE, and *R*^2^, were used to measure the relationship between the actual values and predicted values.  Table 6 summarizes the prediction errors for machine learning to classify the intrusion. It is noted that the KNN algorithm had a robust correlation between the prediction output and classes; the prediction errors of outputs from the KNN algorithm were MSE (0.01449) and (*R*^2^ = 94.17%).

#### 4.1.2. Results of Deep Learning for Binary Classifiers

In this experiment, the LSTM and autoencoder algorithms were applied to classify intrusion as normal and attack.  Table 7 displays the results of deep learning. LSTM achieved good accuracy in detecting intrusion. We observed that the performance of the LSTM algorithm was better than the DAE algorithm. The LSTM approach achieved high accuracy (97.82%).

The performance of the LSTM model to identify intrusion is presented in Figure 5. The accuracy of the LSTM model started at 82% and increased to 98% with 20 epochs. The cross-entropy loss of the LSTM model is shown that validation loss decreased to 0.4.

The training and testing accuracy performance of the DAE algorithm is displayed in Figure 6. The testing accuracy of the DAE algorithm reached 88%. The training loss was 0.114, and the testing loss was 0.106.

### 4.2. Results of Multiple Classifications

In this experiment, 34 major attacks and normal packets were considered in the KDD Cup for detecting malicious attacks. The machine learning algorithms assessed were the QSVM, KNN, linear discriminant, and quadratic discriminant algorithms. The dataset has four major attacks, namely, DoS, Probe, U2R, and R2L attacks. In the KDD Cup dataset, the DoS attack contains 45570 record packets and was divided into 70% for training and 30% for testing.  Table 8 shows the instance values of these attacks. The instance values of each attack are presented in Figure 7.

#### 4.2.1. Machine Learning Algorithm with Multiple Classifications

Table 9 indicates the results obtained using the linear SVM, KNN, linear discriminant, and quadratic discriminant algorithms. From the experimental results, the KNN algorithm achieved 98.28% accuracy for all attacks. Furthermore, the KNN algorithm achieved high accuracy against linear SVM, discriminant, and quadratic discriminant algorithms.

The prediction errors metrics, such as MAE, MSE, RMSE, and *R*^2^, were employed to measure the performance of the machine learning models. The prediction of machine learning, namely, linear SVM, KNN, linear discriminant, and quadratic discriminant algorithms, is summarized in Table 10. The prediction errors of the KNN model were very low (MSE = 0.050), and the correlation between the actual data and prediction was *R*^2^ = 95.22%. This indicates the strength of the KNN model in detecting attacks, namely, DoS, Probe, U2R, and R2L attacks.

#### 4.2.2. Results of Deep Learning for Multiple Classifications

The LSTM and DAE algorithms were applied to detect DoS, Probe, U2R, and R2L attacks.  Table 11 summarizes the results of deep learning. The LSTM model achieved high accuracy compared with the DAE algorithm. The accuracy percentage of LSTM was 97.07% for the classification of multiple attacks.

The performance of LSTM in the testing and training processes is presented in Figure 8. The performance curve shows that the accuracy started from 40% and reached 97.07%, which indicates the reliability of the LSTM model in detecting multiple attacks, and training loss of the LSTM model is decreased to 1.2.

The performance of the autoencoder algorithm is displayed in Figure 9 the cross-entropy loss of the autoencoder algorithm for training and testing is presented, and it is observed that the performance accuracy of the autoencoder algorithm for 200 epochs was not good.

## 5. Discussion

Machine learning is a kind of information-driven approach in which the first step is possible when the data are understood. In the present work, we used data on essential ranking attacks. We presented different ways to apply machine learning techniques to design IDSs for various kinds of data. The various kinds of data represent specific attack behaviors, including the behaviors and activities of the host on the network. Server logs reflect host behaviors and network traffic that represent network behaviors. There are several types of attacks, and each has a particular pattern. Therefore, it is important to select suitable data sources to detect various attacks as per the features of the threat. One of the main features of the DoS attack, for example, is that it is employed to dispatch several packets in a very short period of time, so data stream is ideal for DOS attack detection. A hidden channel includes a data-leaking operation between two different IP addresses and is best for session data discovery.

Developing intelligent systems based on machine learning and deep learning approaches was the main purpose of this study. The KDD Cup dataset is a common network dataset that contains several attacks that were used to evaluate the proposed intelligent model. In this research, we applied various machine learning and deep learning models to design cybersecurity systems in the IoT environment. During the training of the models, we observed the robustness of each model for detection intrusion.

Two experiments were conducted for binary and multiple classification. The main objective was to use the two experiments to design the signature database for detection intrusion. The empirical results of two experiments showed the appropriate algorithms for detecting binary and multiple classes.  Table 12 shows the comparison of machine learning and deep learning models for binary and multiple classes in terms of accuracy. Among the various machine learning and deep learning algorithms, the KNN and LSTM models were found to be appropriate models for detecting intrusion with binary and multiple attacks.

The KNN and LSTM model achieved high accuracy percentages for binary and multiple classification. The performance of KNN showed 98.55% accuracy, where the accuracy of the KNN for classifying multiple classes was 98.28%. Furthermore, the LSTM showed scores of 97.82% and 97.07% for detecting intrusion by binary and multiple classification, respectively.

Receiver operating characteristic (ROC) curves for the LSTM model with binary and multiple classifications are presented in Figure 10. The ROC graphs show the significance of the LSTM model in classifying multiple classes. The *y*-axis represents the true-positive rate of the LSTM model, and the *x*-axis indicates the false-positive rate of LSTM model in detecting normal, DoS, Probe, R2L, and U2R attacks. Overall, the KNN and LSTM models are the best algorithms for detecting attacks of binary and multiple databases.

The comparison of the classification results of the proposed system against existing security system using artificial intelligence approaches is presented in Table 13.

Overall, the proposed system has achieved highest accuracy than eastings systems (97.07%) by using binary classification, whereas the proposed system with multiple classes has achieved 97.82%.

## 6. Conclusion

Considering that Web-based businesses manage exceeding amounts of data and business-related secrets, it is necessary to conduct system movement examinations to achieve appropriate data security.

Therefore, there is a need to develop a smart system to protect IoT networks. Machine learning and deep learning are strategies to detect attacks intelligently. Various machine learning algorithms, namely, QSVM, KNN, linear discriminant, and quadratic discriminant algorithms, were applied, and deep learning algorithms, namely, LSTM and DAE algorithms, were proposed to detect intrusion.

The KDD Cup dataset was employed to test the various machine learning and deep learning algorithms. This dataset has various types of attacks and normal packets. The one-hot encoding method was used to convert four categorical features into numerical features. The dataset has 41 features for consuming training time and improving the performance of the proposed system. The correlation methods were used to select significant features based on high percentage relationships with classes. These selection features were normalized using the min-max normalization method for scaling the data in the same range, which can help to increase the accuracy.

Machine learning and deep learning algorithms were tested with two databases, namely, binary and multiple classifications. Empirical results showed that the KNN and LSTM models achieved high accuracy in binary and multiple classifications. This study offers a comprehensive summary of the proposed algorithms and gives useful insights into the appropriate machine learning and deep learning models for detecting intrusions in IoT systems and any network. The hybrid CNN-LSTM model will be proposed for improving accuracy of the proposed system.[57], [58], [59].

## Figures and Tables

**Figure 1:** Proposed system.

**Figure 2:** Architecture of the LSTM technique.

**Figure 3:** The structure of the autoencoder model for an IDS.

**Figure 4:** Percentage instance values of the KDD Cup data.

**Figure 5:** Performance of LSTM model on binary classification.

**Figure 6:** Performance of DAE model on binary classification.

**Figure 7:** Percentage of values of attacks.

**Figure 8:** Performance of LSTM model on multiple classification.

**Figure 9:** Performance of DAE model on multiple classification.

**Figure 10:** ORC of the LSTM model for multiple classification: (a) normal, (b) DoS attack, (c) probe attack, (d) R2L attack, and (e) U2R attack.

**Table 1:** Feature names of the KDD Cup dataset.

S. No	Feature names
1	Duration
2	Protocol type
3	Service
4	Src-byte
5	Dst-rate
6	Flag
7	Land
8	Wrong_fragment
9	Urgent
10	Hot
11	Nume_faild_login
12	Logged_in
13	Num_compromised
14	Root_shell
15	Su_atte- + mpted
16	Num_root
17	Num_file_creation
18	Num_shells
19	Num_acces_shells
20	Num_outbound_cmds
21	Is_hot_Login
22	Ist_guest_Login
23	Count
24	Serror_rate
25	Rerror-rate
26	Same-Srv-rate
27	Diff-Srv-rate
28	Srv_Count
29	Srv_serror_rate
30	Srv_rerror_rate
31	Srv_Diff_host_rate
32	Dst_host_count
33	Dst_host_srv_count
34	Dst_host_same_srv_count
35	Dst_host_diff_srv_count
36	Dst_host_same_src_port_rate
37	Dst_host_srv_diff_host_rate
38	Dst_host_serror_rate
39	Dst_host_srv_serror_rate
40	Dst_host_rerror_rate
41	Dst_host_srv_rerror_rate

**Table 2:** All types of attacks in the KDD Cup.

Attacks in datasets	Type of attacks in KDD Cup
DoS	Back, Land, Neptune, Pod, Smurf, Teardrop, Mailbomb, Processtable, Udpstor m, Apache2, Worm
Probe	Satan, IPsweep, Nmap, Portsweep, Mscan, Sa int
R2L	Guess_password, Ftp_write, Imap, Phf, Multihop, Warezmaster, Xlock, Xsnoop, Snmpgue, ss, Snmpgetattack, Httptunnel, Sendmail, Named
U2R	Buffer_overflow, Loadmodule Rootkit, Perl, Sqlattack, Xterm, Ps
Attacks in datasets	Type of attacks in NSL-KDD
DoS	Back, Land, Neptune, Pod, Smurf, Teardrop, Mailbomb, Processtable, Udpstor m, Apache2,Worm
Probe	Satan, IPsweep, Nmap, Portsweep, Mscan, Saint
R2L	Guess_password, Ftp_write, Imap, Phf, Multihop, WarezmasterXlock, Xsnoop, Snmpgue, ss, Snmpgetattack, Httptunnel, Sendmail, Named
U2R	Buffer_overflow, Loadmodule Rootkit, Perl, Sqlattack, Xterm, Ps

**Table 3:** Categorical features.

S. No	Feature name
2	Service
3	Flag
6	Protocol type

**Table 4:** Selected features.

No.	Feature name	Correlation (ranking%)
23	count	0.576257
30	srv_serror_rate	0.648135
24	serror_rate	0.650527
38	dst_host_serror_rate	0.651740
39	dst_host_srv_serror_rate	0.654855
12	logged_in	0.690053
36	dst_host_same_srv_rate	0.693525
33	dst_host_srv_count	0.722356
26	same_srv_rate	0.751746

**Table 5:** Performance of binary classifiers to detect intrusion.

Models	Network packets	Accuracy (%)	Precision (%)	Recall (%)	F1 score (%)
QSVM	Normal	95.77	93	92	96
	Attacks		99	99	95

KNN	Normal	98.55	98	99	98
	Attacks		99	98	99

Linear discriminant	Normal	96.77	96	98	97
	Attacks		97	96	97

Quadratic discriminant	Normal	68.91	63	100	77
	Attacks		76	99	86

**Table 6:** Statistical analysis of binary classifiers to predict intrusion.

Models	MAE	MSE	RMSE	*R* ^2^%
QSVM	0.0422	0.0422	0.20	83
KNN	0.0144	0.01449	0.120	94.17
Linear discriminant	0.0323	0.0322	0.1796	87.04
Quadratic discriminant	0.3101	0.310	0.55	13.82

**Table 7:** Results of deep learning in binary classes.

Models	Loss	Accuracy (%)	Precision (%)	Recall (%)	F1 score (%)
LSTM	0.063	97.82	97.25	98.12	97.97
DAE	0.1040	87.40	76.25	98.84	85.71

**Table 8:** Instance values of attacks.

Attacks	#Instance values
Normal	66810
DoS	45570
Probe	11579
R2L	990
U2R	52

**Table 9:** Performance of machine learning algorithms in detecting multiple classes.

Model	Attacks	Accuracy (%)	Precision (%)	Recall (%)	F1 score (%)
Linear SVM	DoS	95.39	95	96	96
	Probe		87	79	83
	R2L		63	62	62
	U2R		0.00	0.00	0.00
	Normal		97	98	98

QSVM	DoS	92.89	96	94	95
	Probe		97	60	74
	R2L		0.00	0.00	0.00
	U2R		0.00	0.000	0.00
	Normal		91	100	95

KNN	DoS	98.28	99	98	99
	Probe		96	97	96
	R2L		91	80	85
	U2R		57	27	36
	Normal		98	99	99

Linear discriminant	DoS	93.18	94	96	95
	Probe		89	73	80
	R2L		33	88	48
	U2R		0.04	60	0.08
	Normal		97	95	96
	DoS	61.79	94	86	90
	Probe		84	28	42
	R2L		0.03	100	0.06
	U2R		0.00	0.00	0.00
	Normal		75	51	61

**Table 10:** Statistical analysis of machine learning for multiple classification.

Models	MAE	MSE	RMSE	*R* ^2^(%)
Linear SVM	0.097	0.274	0.524	92.41
QSVM	0.20	0.648	0.8050	82.81
KNN	0.050	0.172	0.4158	95.22
Linear discriminant	0.145	0.401	0.633	88.90

**Table 11:** Results of deep learning for multiple classification.

Models	Loss	Accuracy (%)	Precision (%)	Recall (%)	F1 score (%)
LSTM model	0.088	97.07	97.34	96.86	97.10
Autoencoder model	0.0676	80.01	80	78.23	88.23

**Table 12:** Significant results of the proposed system.

Model	Accuracy	Experiments
KNN	98.55	Binary classification
LSTM	97.82	Binary classification
KNN	98.28	Multiple classification
LSTM	97.07	Multiple classification

**Table 13:** Comparison results of the proposed system against existing security system using artificial intelligence approaches

Ref.	Model	Datasets	Accuracy %
[56]	SAAE-DNN	NSL-KDD test	87.74%
[57]	ICVAE-DNN	NSL-KDD test	85.97%
[58]	Bagging	NSL-KDD test	90.41%
[59]	GAR-forest	NSL-KDD test	90%
Proposed system	LSTM	NSL-KDD test	97.07% with multiple classification and 97.82 with binary classification

## Data Availability

The data presented in this study are available at https://www.unb.ca/cic/datasets/nsl.html.
